# Neospora caninum SRS2 Protein: Essential Vaccination Targets and Biochemical Features for Next-Generation Vaccine Design

**DOI:** 10.1155/2022/7070144

**Published:** 2022-04-06

**Authors:** Ali Asghari, Bahareh Kordi, Bahman Maleki, Hamidreza Majidiani, Morteza Shams, Razi Naserifar

**Affiliations:** ^1^Department of Medical Parasitology and Mycology, School of Medicine, Shiraz University of Medical Sciences, Shiraz, Iran; ^2^Department of Basic Medical Sciences, Neyshabur University of Medical Sciences, Neyshabur, Iran; ^3^Department of Parasitology, Faculty of Medical Sciences, Tarbiat Modares University, Tehran, Iran; ^4^Zoonotic Diseases Research Center, Ilam University of Medical Sciences, Ilam, Iran

## Abstract

Vaccination is a standout preventive measure to combat neosporosis among cattle herds. The present in silico study was done to evaluate the physicochemical properties and potent immunogenic epitopes of N. caninum SRS2 protein as a possible vaccine candidate. Web-based tools were used to predict physicochemical properties, antigenicity, allergenicity, solubility, posttranslational modification (PTM) sites, transmembrane domains and signal peptide, and secondary and tertiary structures as well as intrinsically disordered regions, followed by identification and screening of potential linear and conformational B-cell epitopes and those peptides having affinity to bind mouse major histocompatibility complex (MHC) and cytotoxic T lymphocyte (CTL). The protein had 401 residues with a molecular weight of 42 kDa, representing aliphatic index of 69.35 (thermotolerant) and GRAVY score of -0.294 (hydrophilic). There were 53 PTM sites without a signal peptide in the sequence. Secondary structure comprised mostly by extended strand, followed by helices and coils. The Ramachandran plot of the refined model showed 90.2%, 8.8%, 0.5%, and 0.5% residues in the favored, additional allowed, generously allowed, and disallowed regions, correspondingly. Additionally, various potential B-cell (linear and conformational), CTL, and MHC-binding epitopes were predicted for N. caninum SRS2. These epitopes could be further utilized in the multiepitope vaccine constructs directed against neosporosis.

## 1. Introduction

Neosporosis is a parasitic disease caused by an intracellular apicomplexan, Neospora caninum (N. caninum) ([1]), with serious sequelae such as reproductive failure in livestock species, particularly in cows [2, 3]. This protozoan also infects rodents, wild ungulates, birds, and marine mammals [4]. The parasite employs two hosts to complete its life cycle, so that dog (Canis familiaris) [5], dingo (Canis dingo) [6], coyote (Canis latrans) [7], and gray wolf (Canis lupus) [8] are definitive hosts, while cattle and buffalo are the most important intermediate hosts [9]. The parasite possesses three distinct infective stages, comprising tachyzoite (acute infection), bradyzoite (chronic infection), and sporozoite (environmental contamination) [10]. Infected canids contaminate the environment through oocyst shedding, being infectious for both canids and herbivores [11]. The parasite is maintained within cattle populations through transplacental transmission, resulting from oocyst ingestion (exogenously) and/or reactivated infection during gestation (endogenously) [12, 13]. In addition to the endemic and/or epidemic abortions in midgestation, there are other factors that economically impact the cattle industry including reduced weight gain in beef calves, decreased milk yield [10], replacing culled animals [14], and the additional costs of veterinary care [15].

Ordinarily, various strategies are proposed to cattle producers in order to reduce infections within herds, including the following: (i) identify and cull infected animals in case of endemic abortions, (ii) prevention of contact between cattle and definitive hosts, hence reducing oocyst contamination, in case of epidemic abortions, (iii) chemotherapy of seropositive animals, and (iv) vaccination protocols [16]. Lack of effective, safe drugs on the one hand and long-time treatment causing the issue of drug residues in food animals on the other hand make treatment troublesome economically [14, 17]. Despite over a decade of research on immunization against N. caninum using various protocols, no commercial vaccine has been developed so far [18]. An ideal vaccination against N. caninum may comply with several issues, encompassing a considerable decline in oocyst shedding by final hosts, reduction of tissue cysts in food animals to avoid transmission via carnivorism, and confining tachyzoite multiplication in pregnant cow to lower the rate of transplacental transmission [16]. Accordingly, such vaccine candidate should stimulate both mucosal and systemic cell-mediated and antibody-dependent components [19]. Thus far, several vaccination strategies using naturally less-virulent isolates and/or attenuated strains have been exploited in cattle and mouse models, showing to be efficacious in spite of safety concerns and production costs [10]. Subunit peptide-based or DNA vaccines are more deeply investigated due to their evident benefits in reduced production, processing, and storage costs along with higher shelf-life and stability [20]. Mostly, those molecules involved in adhesion/invasion processes such as surface antigens (SAGs), microneme (MIC), and rhoptry (ROP) proteins, dense granular (GRA) components, and targets in parasitophorous vacuole membrane (PVM) have been targeted in subunit vaccines [21].

Immunoinformatics is an emerging computer-aided practice for a rational, structure-based vaccine design in a time- and cost-effective manner, which also optimizes biochemical and immunogenic performances [22]. Immunodominant tachyzoite-specific surface antigens such as N. caninum SAG1-related sequence 2 (NcSRS2) have been shown as one of the promising vaccine candidates in murine models, providing protection against lethal challenge or vertical transmission [23–25]. Nevertheless, lack of information on NcSRS2 biochemical features and potential immunogenic epitopes in mouse models directed us to conduct the present in silico study.

## 2. Methods

### 2.1. NcSRS2 Protein Sequence Retrieval

The amino acid sequence of the NcSRS2 protein was retrieved through the UniProtKB database, available at https://www.uniprot.org/, under accession number of Q58L77.

### 2.2. Prediction of Antigenicity, Allergenicity, Solubility, and Physicochemical Characteristics

Antigenicity is a principal characteristic of a vaccine candidate and was evaluated using two web servers: ANTIGENpro (http://scratch.proteomics.ics.uci.edu/) and VaxiJen v2.0 (http://www.ddgpharmfac.net/vaxijen/). The latter is a freely accessible server which predicts on the basis of physicochemical properties of a protein and turns sequences into uniform vectors via auto cross covariance (ACC) approach [26, 27]. Also, ANTIGENpro is a pathogen-independent, alignment-free predictor of antigenicity using a two-stage architecture and five ML algorithms, trained by reactivity information obtained from protein microarray analyses for five pathogens [28]. Three web servers predicted allergenicity, including AlgPred (http://crdd.osdd.net/raghava/algpred/), AllergenFP v1.0 (https://ddgpharmfac.net/AllergenFP/), and AllerTOP v2.0 (http://www.ddg-pharmfac.net/AllerTOP). An alignment-free approach with the Matthews correlation coefficient of 0.759 is employed by AllergenFP v1.0 server [29, 30], while AllerTOP v2.0 exploits several machine learning methods, comprising k-nearest neighbors, cross-variance transformation, and E-descriptors [31]. Moreover, mapping IgE epitopes, MEME (Multiple Em for Motif Elicitation)/MAST (Motif Alignment and Search Tool) allergen motifs were utilized by AlgPred web server to predict allergens [32]. Protein-Sol web server, available at https://proteinsol.manchester.ac.uk/, predicted solubility of NcSRS2 with a threshold score of 0.45 as the population average of the experimental dataset, so higher scores indicate higher protein solubility [33]. Finally, ExPASy ProtParam server (https://web.expasy.org/protparam/) was used to estimate some important physicochemical properties of NcSRS2 such as molecular weight (MW), number of negatively and positively charged residues, aliphatic and instability indices, isoelectric point (pI), half-life, and grand average of hydropathicity (GRAVY) [34, 35].

### 2.3. Prediction of Posttranslational Modification (PTM) Sites

Several PTM sites of NcSRS2 protein were predicted, including serine, threonine, and tyrosine phosphorylation sites by NetPhos 3.1 (http://www.cbs.dtu.dk/services/NetPhos), palmitoylation or acylation sites by CSS-Palm (http://csspalm.biocuckoo.org/), and N-linked and O-linked glycosylation sites by NetNGlyc 1.0 (http://www.cbs.dtu.dk/services/NetNGlyc/) and NetOGlyc 4.0 (http://www.cbs.dtu.dk/services/NetOGlyc/) web servers. “All Asn residues” option was used for NetNGlyc 1.0 prediction, while default parameters were applied to NetOGlyc 4.0 server.

### 2.4. Subcellular Localization, Signal Peptide, and Transmembrane Domain Prediction

For the prediction of subcellular localization, DeepLoc 1.0 server was employed, available at http://www.cbs.dtu.dk/services/DeepLoc/. For transmembrane domain prediction, TMHMM 2.0 server was used, being available at http://www.cbs.dtu.dk/services/TMHMM-2.0. In the following, signal peptide prediction was done using two web servers, including Signal-3L 3.0 (http://www.csbio.sjtu.edu.cn/bioinf/Signal-3L/) and SignalP (http://www.cbs.dtu.dk/services/SignalP/) web servers.

### 2.5. Secondary Structure and Disordered Region Prediction

Prediction of the secondary structure was done by the PSI-blast-based secondary structure PREDiction (PSIPRED) server, which is available at http://bioinf.cs.ucl.ac.uk/psipred/. This server shows many important features in the submitted protein sequence, if available, such as strand, helix, coil, disordered regions, putative domain boundary, membrane interaction, transmembrane helix, extracellular, reentrant helix, and cytoplasmic and signal peptide in both sequence-based and graphical forms [36].

### 2.6. Prediction of the Three-Dimensional (3D) Model, Refinement, and Validations

The homology modelling of the NcSRS2 protein was performed using SWISS-MODEL online tool using default parameters (https://swissmodel.expasy.org/) [37]. In order to establish likely side chains, repacking them and total refinement of the final structure, the GalaxyRefine server (http://galaxy.seoklab.org/cgi-bin/submit.cgi?type=REFINE) was used which provides five refined models for each submitted pdb file, differing on several parameters such as global distance test-high accuracy (GDT-HA), root mean square deviation (RMSD), MolProbity, Clash score, Poor rotamers, and Rama favored [38–40]. Subsequently, the quality improvement of the final structure was evaluated using ProSa-web (*Z*-score) (https://prosa.services.came.sbg.ac.at/prosa.php) [41], ERRAT (quality factor) [42], and PROCHECK (Ramachandran plot analysis) (https://saves.mbi.ucla.edu/) [43].

### 2.7. Prediction of Continuous and Conformational B-Cell Epitopes

A multistep approach was exploited for linear B-cell epitope prediction in NcSRS2. For this aim, a fixed-length prediction (14-mer) with 75% specificity was applied in BCPREDS server (http://ailab.ist.psu.edu/bcpred/predict.html), which uses subsequent kernel (SSK) and support vector machine (SVM) techniques [44–46]. In the next step, cross-validation of the predicted epitopes was accomplished with the outputs of two other web servers, including ABCpred (http://crdd.osdd.net/raghava/abcpred/ABC_submission) [47] and SVMTriP (http://sysbio.unl.edu/SVMTriP/prediction.php) [48]. Those epitopes being shared among outputs of the above servers were selected for further screening regarding antigenicity, allergenicity, and water solubility using VaxiJen v2.0, AllerTOP v2.0, and PepCalc web servers, respectively. Of note, linear B-cell epitopes were, also, predicted by Bcepred server based on different physicochemical parameters such as hydrophobicity, flexibility, accessibility, turns, exposed surface, polarity, and antigenic propensity (http://crdd.osdd.net/raghava/bcepred/bcepred_submission.html). Additionally, conformational B-cell epitopes were predicted using ElliPro tool of the immune epitope database (IEDB) web server (http://tools.iedb.org/ellipro/) [49].

### 2.8. Prediction and Screening of Mouse Major Histocompatibility- (MHC-) Binding Epitopes

All epitope predictions were done using MHC-I (http://tools.iedb.org/mhci/) and MHC-II (http://tools.immuneepitope.org/mhcii) binding epitope prediction tools of IEDB server. Regarding MHC-I-binding epitopes, 8 mouse alleles (H2-Db, H2-Dd, H2-Kb, H2-Kd, H2-Kk, H2-Ld, H-2-Qa1, and H-2-Qa2) were used with subsequent screening in terms of antigenicity, allergenicity, and toxicity through VaxiJen v2.0, AllergenFP v1.0, and ToxinPred (https://webs.iiitd.edu.in/raghava/toxinpred/index.html) servers, respectively. With respect to MHC-II-binding epitopes, 3 mouse alleles (H2-IAb, H2-IAd, and H2-IEd) were employed for epitope prediction, followed by screening regarding antigenicity, allergenicity, toxicity, IFN-*γ,* and IL-4 induction using VaxiJen v2.0, AllergenFP v1.0, ToxinPred, IFNepitope (https://webs.iiitd.edu.in/raghava/ifnepitope/application.php), and IL4-pred (https://webs.iiitd.edu.in/raghava/il4pred/design.php) web servers, correspondingly.

### 2.9. Prediction and Screening of Cytotoxic T-Lymphocyte (CTL) Epitopes

Top 10 CTL epitopes of NcSRS2 protein were predicted using CTLpred web server (https://bio.tools/ctlpred), followed by screening regarding antigenicity, allergenicity, and hydrophobicity using VaxiJen v2.0, AllergenFP v1.0, and peptide2 (https://www.peptide2.com/N_peptide_hydrophobicity_hydrophilicity.php) web servers, respectively.

## 3. Results

### 3.1. General Characteristics of the NcSRS2 Protein

A considerably high antigenic index was predicted for this protein, as substantiated by a VaxiJen score of 0.8286 and ANTIGENpro score of 0.966227. Based on the findings from three web servers, no allergenicity, IgE epitopes, and MEME/MAST motifs were found for NcSRS2 protein. High solubility (over 0.45) was, also, predicted by Protein-Sol server with a solubility score of 0.523 (Figure 1). This protein possessed 401 amino acid residues, with a MW of 42009.93 kilo Dalton (kDa) and 45 and 35 negatively (Asp+Glu) and positively charged (Arg+Lys) residues. The extinction coefficients at 280 nm measured in water was 30910 (assuming all pairs form cystines) and 29910 (assuming all Cys residues are reduced) M^−1^ cm^−1^. The estimated half-life was 30 hours in mammalian reticulocytes (in vitro), >20 hours in yeast (in vivo), and >10 hours in Escherichia coli (in vivo). The protein was rendered as unstable, since instability index was computed to be 49.24. Moreover, aliphatic index, GRAVY score, and pI of the protein were calculated to be 69.35, -0.294, and 5.28, respectively.

### 3.2. Prediction of PTM Sites, Subcellular Localization, Transmembrane Domain, and Signal Peptide

In total, 36 phosphorylation sites were present in the NcSRS2 protein using NetPhos server, encompassing 21 serine, 11 tyrosine, and 4 threonine sites. Also, a palmitoylation site at position 6 was found with a score of 36.903 using CSS-Palm server. In addition, NetNGlyc and NetOGlyc web servers predicted 3 and 14 N-glycosylation and O-glycosylation sites in the examined protein, respectively. A putative transmembrane domain was predicted for this protein, as demonstrated by TMHMM server. Outputs of the Signal-3L server (reliability 0.347) and SignalP web tools (Other: 0.6873) showed no traits of a signal peptide in NcSRS2 protein. DeepLoc subcellular localization analysis revealed that NcSRS2 is probably a soluble (likelihood: 0.4508), extracellular protein (likelihood: 0.3435) with membrane localization (likelihood: 0.5492) (Figure 1).

### 3.3. Secondary Structure Prediction and Disordered Regions

Based on the PSIPRED server analysis with high confidence in most parts, extended strand was the predominant secondary structure in the NcSRS2 protein, followed by helices and coils. Also, 61 residues at N-terminal and 93 residues at C-terminal were intrinsically disordered regions in the protein (Figure 2).

### 3.4. 3D Structure Modelling, Refinement, and Validations

Two models were built by SWISS-MODEL server, among which a monomer model (template: 2 × 28.1. A) with high coverage and sequence identity of 17.29% was selected for further analysis (Figure 3(a)). This model belonged to sporozoite-specific SAG protein. In the following, GalaxyRefine server provided five models, among which model number five with the following parameters was chosen as the best-fit refined model: GDT-HA: 0.9764, RMSD: 0.352, MolProbity: 2.056, Clash score: 22.0, Poor rotamers: 1.4, and Rama favored: 97.5. Finally, the quality of the refined model, as compared with the crude model, was evaluated using three web servers. The Z-score and quality factor of the crude model were -8.07 and 68.493, which were improved to -8.27 and 88.584 after refinement, respectively. The Ramachandran plot analysis of the crude model showed that 82.9%, 15.6%, 1.5%, and 0.0% of residues are assigned to most favored, additional allowed, generously allowed, and disallowed areas, respectively. Upon refinement, they were improved to 90.2%, 8.8%, 0.5%, and 0.5%, correspondingly (Figures 3(b) and 3(c)).

### 3.5. Linear and Conformational B-Cell Epitopes

A cross-validation method was applied to find shared linear B-cell epitopes. Accordingly, 9 epitopes were found and subsequent screening showed that only two epitopes are potentially antigenic and nonallergenic with good water solubility, including “ECKERPYSAVFPGF” and “GPDGKAFPDDY” (Table 1). Moreover, several continuous B-cell epitopes of NcSRS2 protein were determined on the basis of various physicochemical parameters using Bcepred web server (Table 2). Also, ElliPro tool of the IEDB analysis resource demonstrated that there are 4 conformational B-cell epitopes in this protein with the following lengths and scores: (i) 34 residues, score: 0.713; (ii) 46 residues, score: 0.705; (iii) 42 residues, score: 0.666; and (iv) 16 residues, score: 0.657 (Figure 4).

### 3.6. Prediction of Mouse MHC-Binding and CTL Epitopes

For each mouse MHC-I (H2-Db, H2-Dd, H2-Kb, H2-Kd, H2-Kk, H2-Ld, H-2-Qa1, and H-2-Qa2) and MHC-II allele (H2-IAb, H2-IAd, and H2-IEd), five and six epitopes having the lowest percentile rank (higher affinity) were chosen, respectively, which then subjected to screening in terms of antigenicity, allergenicity, toxicity (MHC-I and MHC-II), and IFN-*γ*/IL-4 induction (MHC-II). Regarding mouse MHC-I-binding epitopes, seven epitopes had the highest antigenicity score, while they were nonallergenic and nontoxic, including “ITVNPENNGVTL,” “GHPDDKQVTCVV,” “VAHCAYSSNVRL,” “TVNPENNGVTLI,” “SPVLRGDACDEL,” “SAVFPGFSSSFW,” and “KEWVTGTLQQGI” (Table 3). Furthermore, three mouse MHC-II-binding epitopes were capable to induce IFN-*γ* with high antigenicity and without allergenic and toxic traits, comprising “HCAYSSNVRLRPITV,” “AHCAYSSNVRLRPIT,” and “VAHCAYSSNVRLRPI” (Table 4). Also, top ten CTL epitopes were predicted using CTLpred server, among which 4 epitopes possessed highest antigenicity and hydrophobicity and without allergenicity, encompassing “AYSSNVRLR,” “LRGDACDEL,” “RESEVIGQV,” and “SEDDGLIVC” (Table 5).

## 4. Discussion

First insights into the immunobiology of the apicomplexan parasite, N. caninum, in cattle and dogs were revealed during 1999 to 2003 [18], leading to the initial vaccination approaches in the mouse model [25] as well as cattle as target species [50]. In parallel with the deciphering the parasite biology and identification of parasitic antigens, more researches on N. caninum vaccination were flourished during last decade, using novel antigens and different immunization platforms. Having no live component, subunit vaccines represent no risk of disease induction; hence, they are mostly focused for a safe vaccination, usually accompanied by an adjuvant as an immune promoter compound [22]. Innovative technology-oriented methods such as reverse vaccinology and immunomics have facilitated the appropriate screening and selection of potential antigenic targets among multiple proteins and assisted us to deeply explore and highlight the immunogenic epitopes within the amino acid sequence of a given protein [22]. Until now, several surface expressed and excretory/secretory proteins have been recognized as vaccine candidates [23, 51–54], while in silico analysis of such proteins and identification of potential immunogenic epitopes was lacking. The present in silico study was performed to highlight several important biochemical properties of the NcSRS2 protein and to identify novel immunogenic epitopes for future vaccination and/or diagnostic purposes in the context of multiepitope protein constructs.

The SRS protein superfamily of N. caninum contains about 227 genes and 52 pseudogenes [55, 56], substantially higher than Toxoplasma gondii (T. gondii) strains [57]. Neospora caninum SAG1 and SRS2 are principal immunodominant surface antigens in tachyzoites, which mediate an initial low-affinity, reversible adhesion to the host cell prior to invasion [23]. Previously, several vaccination studies were done using NcSRS2 alone and/or combined with other parasitic antigens. A satisfactory transplacental protection was obtained upon immunization with recombinant NcSRS2 expressed using a viral vector (vaccinia virus) [25]. The application of NcSRS2 immune-stimulating complexes (ISCOMS) in different formulations reduced the cerebral parasite burden and induced specific antibody responses [58, 59]. Mice vaccinated with a set of antigens such as NcGRA6, NcGRA7, NcMIC1, and NcSRS2 expressed in a bacterial vector (Brucella abortus) provided complete protection against acute disease [60]. Another study using N. caninum cyclophilin-a potent IFN-*γ* inducer and NcSRS2 showed to be highly efficacious in antibody production and inhibiting cerebral infection [61]. It seems that vaccination with NcSRS2 may play a crucial role in protection against cerebral parasites, though it demands further experimental evidences. Altogether, these findings highlight the importance of NcSRS2 as a promising vaccine candidate. “From a biochemical standpoint, a protein is represented in four structural levels, comprising: (i) amino acid sequences as primary structure, (ii) a native spatial form due to main chain atoms (*α*-helix and *β*-fold) as secondary structure, (iii) potential spatial model as a 3D model or tertiary structure, and (iv) number and position of multi-fold subunits in a multi-subunit collection of a protein as quaternary structure” [62–64]. In the first step of this study, we characterized general biochemical features of the protein. It was found that NcSRS2 is a highly antigenic molecule (VaxiJen score: 0.8286, ANTIGENpro: 0.966227), while no allergenic, MEME/MAST motifs and IgE epitopes were found within the sequence; the antigenicity of the NcSRS2 was even higher than the immunodominant molecule, NsSAG1 (VaxiJen score: 0.6278) [65]. High protein solubility was calculated for NcSRS2, with Protein-Sol score of 0.523, similar to NcSAG1 with a solubility of 0.620 [65]. The MW of the NcSRS2 was 42 kDa (those proteins over 5-10 kDa are potent immunogens) [66–68], which is beneficial for SDS-PAGE and western blot analyses. Instability index of over 40 renders the protein to be unstable in vitro, as substantiated by instability score of 49.24. Moreover, this protein was moderately thermotolerant in a wide range of temperatures (aliphatic index: 69.35) and showed to be somehow hydrophilic in nature (GRAVY score: -0.294), contrary to NcSAG1 (GRAVY: 0.031) [65]. The speculated pI for this protein was estimated as relatively acidic in nature (5.28), being advantageous for purification purposes in ion-exchange chromatography and isoelectric focusing. In contrast, the pI of NsSAG1 protein was estimated as 7.89 [65]. Altogether, such preliminary information may be required for future wet studies using NcSRS2. With 36 regions, phosphorylation was the predominant PTM site in NcSRS2 protein, followed by O-glycosylation (14 regions), N-glycosylation (3 regions), and palmitoylation sites (one region). In total, these PTM regions are crucial in the recombinant production process of the proteins, so that eukaryotic expression systems (yeast, insect, or mammalian) are more preferred in comparison to bacterial hosts [69]. The presence of a signal peptide demonstrates that a synthesized protein could be destined towards several pathways, including excretory-secretory, virulence factor, or surface proteins [70]. Accordingly, based on the results from Signal-3L and SignalP web servers, no signal peptide was present in the sequence. PSIPRED server demonstrated that extended strands are the most prevalent secondary structure in the NcSRS2 protein, followed by helices and coils; inevitably, the protein conformation is maintained and protected during molecular interactions using such internally located structures [71]. Notably, it was found that 61 residues and 93 residues at N-terminal and C-terminal of the sequence are disordered. Disordered proteins are highly abundant, mostly dedicated to regulatory functions and molecular signaling. Supposedly, these regions are likely immunological targets for antibodies; hence, they seem to be important in vaccination studies [72]. For 3D homology modelling, SWISS-MODEL server was employed, which predicted a monomer model with high coverage and 17.29% identity. Actually, the protein possesses a homodimeric form with two domains (D1 and D2) linked by a cysteine bridge (disulfide bonds) as a well-known representative in SRS proteins of T. gondii and N. caninum [73–76]. Such a marvelous, conserved folding pattern in SRS antigens may be pivotal for their biological function as they potentially couple with sulphated proteoglycan-binding site in target cell receptors [73, 76, 77]. In the following, the 3D model was further subjected to refinement and validations. Based on the ERRAT, ProSa-web, and PROCHECK analyses, it was shown that the quality of the refined model was enhanced after refinement, in comparison with the crude model.

During early N. caninum infection, a CD_4_^+^ Th1 polarization is a predominant response, leading to IL12-dependent IFN-*γ* upsurge as a protective immune response [78]. Such specific T-cells are highly vital for protection against the infection in mice. Humoral responses, also, play a critical role in protection mostly biased by IgG2a antibody response in mice. Although cattle is the target species for vaccination studies against neosporosis, mouse models are more accessible and affordable for such purposes [78]. As well, utilization of murine models is a basic step for evaluation of the efficacy of vaccination against neosporosis and toxoplasmosis; accordingly, we premised our immunoinformatics analyses on mouse MHC-I- and MHC-II-binding epitopes. Based on this, several web servers were employed in the present study to accurately predict and screen the potential immunogenic epitopes in NcSRS2. A multistep approach was conducted to screen linear B-cell epitopes using six web servers, three for identification of shared epitopes (BCPREDS, ABCpred, and SVMTriP) and three for screening phase (VaxiJen, AllerTOP, and PepCalc). Only two epitopes qualified to be a potential immunogenic epitope, including “ECKERPYSAVFPGF” and “GPDGKAFPDDY.” Conformational B-cell epitopes, also, have a remarkable role in the quality of antigen-antibody interactions. Thereby, we predicted these epitopes in the NcSRS2 protein. The results showed 4 conformational epitopes by the length of 34, 46, 42, and 16 residues, respectively, and qualifying scores of 0.713, 0.705, 0.666, and 0.657. Furthermore, since antigen presentation is highly important for T-cell priming, those epitopes with specific affinity to bind mouse MHC molecules were predicted using IEDB server. With respect to MHC-I-binding epitopes, seven peptides were shown to be highly antigenic, nonallergenic, and nontoxic, including “ITVNPENNGVTL,” “GHPDDKQVTCVV,” “VAHCAYSSNVRL,” “TVNPENNGVTLI,” “SPVLRGDACDEL,” “SAVFPGFSSSFW,” and “KEWVTGTLQQGI.” Also, three MHC-II-binding peptides “HCAYSSNVRLRPITV,” “AHCAYSSNVRLRPIT,” and “VAHCAYSSNVRLRPI” were potent IFN-*γ* inducers, highly antigenic epitopes predicted in the context of H2-IEd mouse allele. Previously, Staska et al. [79] showed that residues located at 133-155 of NcSRS2 protein, including most of the above MHC-I and MHC-II epitopes predicted in our study, may represent an epitope cluster, and they are potential IFN-*γ* inducers in T-lymphocyte cell lines from N. caninum-infected cattle [79]. In this sense, a recently published paper demonstrated that NcSRS2 lipopeptides formulated with Freund's adjuvant encompassing amino acids 77 to 95 and 133 to 155 could robustly induce IFN-*γ*-secreting T-lymphocytes as well as specific serum antibody responses in immunized cattle [80]. Future vaccinology studies in both mouse and cattle should, therefore, particularly emphasize on this section of the protein. However, other residues also should not be neglected to design more efficacious vaccine candidates. Finally, among the top ten CTL epitopes predicted for NcSRS2 protein in our study, only four “AYSSNVRLR,” “LRGDACDEL,” “RESEVIGQV,” and “SEDDGLIVC” qualified as the potential immunogenic epitopes. Altogether, all of these epitopes could be further supplied in the multiepitope vaccine constructs and/or diagnostic polypeptides and be evaluated in the context of wet experimental methods.

## 5. Conclusion

Neospora caninum infection is a global threat to the cattle industry by inflicting reproductive failure and endemic/epidemic abortions. Therefore, there is an increasing need to recognize novel vaccine candidates to be used in the context of unprecedented immunization platforms. The interdisciplinary branch of science, bioinformatics, assist us to characterize the physicochemical features of a protein, to spot highly immunodominant epitopic regions, and to engineer a more rational vaccine design. The apicomplexan SRS proteins are exclusively immunodominant antigens with particular implication in diagnostic tools and/or vaccine candidates. The present in silico study highlighted the most important biophysical characteristics and novel B-cell, MHC-binding, and CTL epitopes of NcSRS2 protein using a set of immunoinformatics servers. This homodimeric protein possesses several potential antigenic epitopes, particularly in 133 to 155 residues, being capable to induce humoral and cellular responses and could be directed towards immunization studies alone or combined with other dominant N. caninum antigens.

## Figures and Tables

**Figure 1:** Computed solubility (a) and subcellular localization (b) of the NcSRS2 protein.

**Figure 2:** Secondary structure prediction by PSIPRED server showing the predominance of extended strand.

**Figure 3:** NcSRS2 protein homology modelling and refinement validation using the Ramachandran analysis. (a) The final tertiary model of NcSRS2 provided by SWISS-MODEL web server, as shown in ribbon. (b) Ramachandran plot analysis of the crude model using PROCHECK demonstrated that 82.9%, 15.6%, 1.5%, and 0.0% of residues are assigned to most favored, additional allowed, generously allowed, and disallowed areas, respectively. (c) Upon refinement, these parameters were improved to 90.2%, 8.8%, 0.5%, and 0.5%, respectively.

**Figure 4:** Predicted conformational B-cell epitopes of NcSRS2 using ElliPro tool of IEDB server. Length and score of each epitope were as follows: (1) 34 residues, score: 0.713; (2) 46 residues, score: 0.705; (3) 42 residues, score: 0.666; and (4) 16 residues, score: 0.657.

**Table 1:** The final screening of shared linear B-cell epitopes from N. caninum SRS2.

Shared B-cell epitopes	VaxiJen antigenicity score	AllergenFP allergenicity prediction	PepCalc water solubility prediction
VAKPAGAGSN	1.1244	Yes	Good
ECKERPYSAVFPGF∗	1.3682	No	Good
VNRSVSVFA	0.0040	Yes	Poor
VALVYDSQHSIT	0.6158	No	Poor
FSSSFWTGEASGVA	1.2775	No	Poor
KADAACFAKLSASQ	-0.0772	No	Good
GPDGKAFPDDY∗	1.6063	No	Good
NNGVTLICGPD	-0.3786	No	Poor
KAGKNVCLL	0.4119	Yes	Good

∗ indicates antigenic, non-allergenic epitopes with potential good water solubility.

**Table 2:** Specific B-cell linear epitopes of N. caninum SRS2 based on different physicochemical parameters predicted by the Bcepred web server.

Physicochemical parameter	Linear B-cell epitopes
Hydrophilicity	FKSENEKF, PKQGNADQ, ACDGGTP, VCNESDGEDECEKNAA, GCKAGKN, VQSRESEV, TVNPENNGV, CGPDGKA, ELDECKERP, GCTGHPDDKQVTC, GAGSNPGGGSQPDQSSEKRDGEQVNKGKPPTGGSGGATTGKQNASQNAKDKGETGGENGDSPV, and RGDACDE

Flexibility	LTAKSVN, APFKSEN, IVCNESDGE, NVYVQSRES, ITVNPEN, TELDECK, AVFPGFS, and AGAGSNPGGGSQPDQSSEKRDGEQVNKGKPPTGGSGGATTGKQNASQNAKDKGETGGENGD

Accessibility	VVRRKADAA, TAKSVNRS, APFKSENEKFTC, PKQGNADQ, KLLSEDD, NESDGEDECEKNA, LPGAKKEWVTG, TIPDEHYPATSKA, YVQSRESEV, SNVRLRP, TVNPENNGV, KAFPDDYMNHH, TELDECKERPYSAV, LTIPKDQFPST, TGHPDDKQVT, GGSQPDQSSEKRDGEQVNKGKPPTGGS, and ATTGKQNASQNAKDKGETGGENGDSP

Turns	NPENNGV, DYMNHHCTE

Exposed surface	FKSENEKF, EDECEKN, DECKERPYSA, PDQSSEKRDGEQVNKGKPPT, and KQNASQNAKDKGE

Polarity	HACVVRRKADAA, PFKSENEKFTC, KLLSEDD, NESDGEDECEKNAA, PGAKKEWVTG, VQSRESEVIG, DDYMNHHCTELDECKERPYSA, TGHPDDKQV, NIEEVAK, DQSSEKRDGEQVNKGK, NAKDKGETG, and RGDACDE

Antigenic propensity	VNRSVSV, LLFGVVLAVGV, FTCLPKQ, LVYDSQH, PLPSKLLS, DDGLIVCNES, PLSTFLP, GKNVCLLNVYVQSRESEVIGQV, NGVTLICGP, QTIYLGCTG, DKQVTCVVPVNIE, and CDELPSY

**Table 3:** Prediction of mouse MHC-I-binding epitopes of N. caninum SRS2 using IEDB server followed by antigenicity, allergenicity, and toxicity screening.

Mouse MHC-I alleles	Position	T-cell peptide	Percentile rank	VaxiJen antigenicity score	AllergenFP allergenicity prediction	ToxinPred toxicity prediction
H2-Db	24-35	ITVNPENNGVTL∗	0.61	1.3534	No	Nontoxin
	44-55	VGCKAGKNVCLL	5.4	0.2220	Yes	Toxin
	4-15	YSAVFPGFSSSF	5.4	0.4492	No	Nontoxin
	47-58	KAGKNVCLLNVY	6.7	-0.0962	No	Toxin
	10-21	VAHCAYSSNVRL	7.7	1.5329	No	Nontoxin

H2-Dd	4-15	YSAVFPGFSSSF	0.58	0.4492	No	Nontoxin
	6-17	LSTFLPGAKKEW	4.7	0.0692	Yes	Nontoxin
	48-59	GHPDDKQVTCVV∗	4.7	1.7670	No	Nontoxin
	24-35	ITVNPENNGVTL	5.5	1.3534	No	Nontoxin
	26-37	VNPENNGVTLIC	6.7	1.0295	No	Nontoxin

H2-Kb	10-21	VAHCAYSSNVRL∗	2.7	1.5329	No	Nontoxin
	31-42	SVNRSVSVFALL	4.0	-0.3061	No	Toxin
	4-15	YSAVFPGFSSSF	5.1	0.4492	No	Nontoxin
	6-17	AVFPGFSSSFWT	7.9	0.8884	No	Nontoxin
	32-43	VNRSVSVFALLF	9.3	0.1617	No	Nontoxin

H2-Kd	24-35	SYVALSAASLTA	2.9	0.4534	No	Nontoxin
	4-15	YSAVFPGFSSSF	6.0	0.4492	No	Nontoxin
	33-44	EHYPATSKAFRV	6.1	0.3313	No	Nontoxin
	33-44	DQFPSTAQTIYL	6.6	-0.0877	No	Toxin
	31-42	PKDQFPSTAQTI	7.0	0.1665	No	Nontoxin

H2-Kk	25-36	TVNPENNGVTLI∗	1.4	0.9366	No	Nontoxin
	17-28	DACDELPSYVAL	1.6	0.1381	Yes	Nontoxin
	3-14	ETGGENGDSPVL	3.1	1.1581	Yes	Nontoxin
	33-44	DQFPSTAQTIYL	3.9	-0.0877	No	Toxin
	15-26	KEWVTGTLQQGI	4.9	1.2743	No	Nontoxin

H2-Ld	36-47	LPSKLLSEDDGL	0.42	0.0641	Yes	Nontoxin
	22-33	LPSYVALSAASL	0.92	0.2773	No	Nontoxin
	24-35	ITVNPENNGVTL	1.2	1.3534	No	Nontoxin
	11-22	SPVLRGDACDEL∗	1.3	1.3596	No	Nontoxin
	22-33	RPITVNPENNGV	1.7	1.3057	Yes	Nontoxin

H-2-Qa1	4-15	YSAVFPGFSSSF	2.1	0.4492	No	Nontoxin
	17-28	ALVYDSQHSITF	3.3	0.4102	No	Nontoxin
	33-44	VTLICGPDGKAF	5.1	0.4982	Yes	Nontoxin
	24-35	ITVNPENNGVTL	5.4	1.3534	No	Nontoxin
	5-16	SAVFPGFSSSFW∗	5.4	1.0065	No	Nontoxin

H-2-Qa2	25-36	TVNPENNGVTLI	2.5	0.9366	No	Nontoxin
	15-26	KEWVTGTLQQGI∗	3.1	1.2743	No	Nontoxin
	17-28	ALVYDSQHSITF	3.1	0.4102	No	Nontoxin
	33-44	DQFPSTAQTIYL	4.1	-0.0877	No	Toxin
	3-14	ETGGENGDSPVL	5.3	1.1581	Yes	Nontoxin

∗ indicates potential high-ranked, antigenic, nonallergenic, and nontoxic epitopes.

**Table 4:** Prediction of mouse MHC-II-binding epitopes of N. caninum SRS2 using IEDB server followed by screening for antigenicity, allergenicity, toxicity, and IFN-*γ*/IL-4 induction.

Mouse MHC-II alleles	Position	T-cell peptide	Percentile rank	VaxiJen antigenicity score	AllergenFP allergenicity prediction	ToxinPred toxicity prediction	IFN-*γ* induction	IL-4 induction
H2-IAb	23-37	PSYVALSAASLTATA	1.1	0.4796	No	Nontoxin	Positive	Negative
	22-36	LPSYVALSAASLTAT	1.21	0.3898	No	Nontoxin	Positive	Negative
	24-38	SYVALSAASLTATAI	1.41	0.4271	No	Nontoxin	Positive	Negative
	21-35	ELPSYVALSAASLTA	1.5	0.4580	No	Nontoxin	Negative	Negative
	25-39	YVALSAASLTATAIF	1.76	0.3833	No	Nontoxin	Negative	Negative
	2-34	DELPSYVALSAASLT	1.85	0.2164	No	Nontoxin	Negative	Negative

H2-IAd	20-34	DELPSYVALSAASLT	0.64	0.2164	No	Nontoxin	Negative	Negative
	21-35	ELPSYVALSAASLTA	0.73	0.4580	No	Nontoxin	Negative	Negative
	22-36	LPSYVALSAASLTAT	0.73	0.3898	No	Nontoxin	Positive	Negative
	23-37	PSYVALSAASLTATA	0.98	0.4796	No	Nontoxin	Positive	Negative
	24-38	SYVALSAASLTATAI	1.39	0.4271	No	Nontoxin	Positive	Negative
	19-33	CDELPSYVALSAASL	1.59	0.3479	No	Nontoxin	Negative	Positive

H2-IEd	1-15	MATHACVVRRKADAA	1.99	-0.3581	No	Nontoxin	Negative	Negative
	2-16	ATHACVVRRKADAAC	2.75	-0.5192	Yes	Nontoxin	Negative	Positive
	12-26	HCAYSSNVRLRPITV∗	3.00	1.3421	No	Nontoxin	Positive	Negative
	11-25	AHCAYSSNVRLRPIT∗	3.35	1.4654	No	Nontoxin	Positive	Negative
	3-17	THACVVRRKADAACF	3.9	-0.6533	Yes	Nontoxin	Negative	Positive
	10-24	VAHCAYSSNVRLRPI∗	4.1	1.3060	No	Nontoxin	Positive	Negative

∗ indicates high-ranked, antigenic, and nonallergenic epitopes with potential IFN-*γ* induction.

**Table 5:** Prediction of top ten cytotoxic T-lymphocyte (CTL) epitopes of N. caninum SRS2 using CTLpred web server with antigenicity, allergenicity, and hydrophobicity screening.

Rank	Start position	Peptide sequence	Score (ANN/SVM)	VaxiJen antigenicity score	AllergenFP allergenicity prediction	Hydrophobicity (%)
1	194	AYSSNVRLR∗	0.57/1.3921456	1.6339	No	33.33
2	70	GNADQWVAL	0.57/1.1068306	0.4913	No	55.56
3	374	LRGDACDEL∗	0.90/0.57070616	1.5932	No	33.33
4	182	RESEVIGQV∗	0.61/0.78029309	1.5955	No	33.33
5	228	YMNHHCTEL	0.65/0.73549537	0.4257	No	22.22
6	127	STFLPGAKK	0.93/0.44198631	0.1985	Yes	44.44
7	1	MATHACVVR	0.82/0.53762368	0.0049	No	55.56
8	328	KRDGEQVNK	0.82/0.44522211	1.3420	No	11.11
9	28	TAKSVNRSV	0.61/0.65066346	0.2242	No	33.33
10	102	SEDDGLIVC∗	0.65/0.59971526	1.9440	No	33.33

∗ indicates antigenic, nonallergenic, and hydrophobic CTL epitopes.

## Data Availability

The data used to support the findings of this study are available from the corresponding author upon request.
